# Value of a Signature of Immune-Related Genes in Predicting the Prognosis of Melanoma and Its Responses to Immune Checkpoint Blocker Therapies

This article has been retracted.

**DOI:** 10.1155/2022/9633416

**Published:** 2022-06-20

**Authors:** Bo Yuan, Linlin Miao, Disen Mei, Lingzhi Li, Qiongyan Zhou, Dong Dong, Songting Wang, Xiaoxia Zhu, Suling Xu

**Affiliations:** ^1^Dermatology Department, The Affiliated Hospital of Medical School, Ningbo University, 247 Renmin Road, Jiangbei District, Ningbo 315020, China; ^2^Surgery Department, School of Medicine, Ningbo University, No. 818, Fenghua Road, Jiangbei District, Ningbo 315210, China; ^3^Basic Medicine Experiment Center, School of Medicine, Ningbo University, 818 Fenghua Road, Jiangbei District, Ningbo 315211, China; ^4^Plastic and Reconstructive Surgery Department, The Affiliated Hospital of Medical School, Ningbo University, 247 Renmin Road, Jiangbei District, Ningbo 315020, China

## Abstract

Melanoma is becoming increasingly common worldwide, with high rates of transformation into malignancy compared to other skin lesions. The prognosis of patients with melanoma at an advanced stage is highly unsatisfying despite the development of immunotherapy, target therapy, or combinative therapy. The major barrier to exploiting immune checkpoint therapies and achieving the best benefits clinically is resistance that can easily develop if regimens are not selected appropriately. In this study, we investigated the possibility of using immune-related genes to predict patient survival and their responses to immune checkpoint blocker therapies with the expression profiles available at The Cancer Genome Atlas (TCGA) Program plus expression data from the Gene Expression Omnibus (GEO) for validation. A five gene signature that is highly correlated with the local infiltration of cytotoxic lymphocytes in the tumor microenvironment was identified, and a scoring model was developed with stepwise regression after multivariate Cox analyses. The score calculated strongly correlates with Breslow depth, and this model effectively predicts the prognosis of patients with melanoma, whether primary or metastasized. It also depicts the heterogenous immune-related nature of melanoma by revealing different predicted responses to immune checkpoint blocker therapies through its correlation to tumor immune dysfunction and exclusion (TIDE) score.

## 1. Introduction

Melanoma develops when melanocytes undergo malignant transformation [1] and can occur in multiple sites of the body such as in the eyes, sinuses, the digestive tracts, and even meninges. The most common site melanoma arises from is in the skin, and even though melanoma is much less frequently seen than other types of skin cancers, the cutaneous form of melanoma causes the majority of deaths related to skin cancer in developed countries, because if not identified and intervened promptly, it is much more likely to spread and metastasize. Varying effectiveness of early screening and different levels of accessibility to treatments in a timely fashion both contributed to the divergent results of overall survival.

Years ago, patients suffering from melanoma with distant metastases had an overall 5-year survival rate below 10% [2]. One decade later, thanks to the drastic advancement in the strategies for treating melanoma, patients receiving combinative targeted therapies and/or immune blocker therapies enjoy a greater chance of surviving longer [3–5]. However, even though remarkable clinical benefits have been witnessed in the treatments of melanoma, melanoma still poses a great cancer burden globally. The incidence rates of melanoma have increased by 170% from 1990 to 2019, and deaths resulting from it also have increased by 90% worldwide [6]. A considerable loss of life in years is caused by the cutaneous subtype of melanoma, one of the most common cancers in young adults in their late 20s or early 30s, which calls for the urgent need for a better therapeutic regimen and hopefully, more effective intervention at a much earlier stage in the development of this disease.

Despite the malignant nature of melanoma, spontaneous regressions of even metastatic melanoma have been reported with rates from 2.7 to 15% [7, 8], so researchers have been very intrigued by exploring the crosstalk between melanoma cells and the immune system. In fact, this interaction between malignant melanocytes and other components present in the tumor microenvironment turns out to be a crucial part in the proliferation and the progression of melanocytes [9–11]. The idea of immunosurveillance has been brought up for more than 50 years [12], but this concept and immunotherapies generated out of it were widely accepted until recently. The immune system constantly checks and differentiates what belongs to “oneself” and what is “foreign.” To initiate sequences of cytotoxic effects and eliminate malignant melanocytes, immune cells must first recognize what is not “self.” Therefore, one crucial method malignant melanocytes exploit to escape from the immune system is through expressing ligands for immune checkpoint proteins such as programmed cell death proteins (PDCDs, or PDs) and cytotoxic T lymphocyte-associated antigens (CTLAs). By binding to their receptors expressed on lymphocytes, the inhibitory effects on the immune system and the refrainment of immune cells can help malignant cells survive [13]. Originally, this suppressing effect is supposed to be generated to maintain self-tolerance and limit inflammation in normal tissue [14–16]. Immunotherapies involving the blockade of CTLA-4 [1, 17] and PD-1 or PD-L1 [18–24] have greatly improved the status and furthered the survival of patients with advanced melanoma.

Nevertheless, it remains challenging to reveal the immune-related nature of melanoma. The precise mechanism underlying the show played by immune cells, especially cytotoxic lymphocytes and melanocytes, stays unknown. It is still challenging to predict patients' responses to the immune checkpoint blockade therapies considering the complexity of the immune system and the lack of long-term follow-ups in large cohorts. Therefore, with available expression profiles in the Cancer Atlas Program and Gene Expression Omnibus, we conducted a series of bioinformatical analyses and identified a signature of 5 immune-related genes that could consistently predict the prognosis of melanoma (advanced stage or not). A risk score calculated based on a model built upon this signature is also capable of depicting the dysregulated expression of immune checkpoint genes as well as responses to immune checkpoint blocker therapies.

## 2. Materials and Methods

### 2.1. Identification of Immune-Related Differentially Expressed Genes (IR-DEGs) That Were Associated with Cytotoxic Lymphocyte Infiltration

#### 2.1.1. Source of Data

Both expression profiles from the skin cutaneous melanoma project of The Cancer Genome Atlas Program (TCGA-SKM) and the GSE53118 (acquired from Gene Expression Omnibus (GEO) at https://www.ncbi.nlm.nih.gov/geo) were exploited in this study. Two cohorts consisting of only primary melanoma samples were randomly selected from the main TCGA-SKM cohort. One of them included 30 samples while the other included 69 samples. Different cohorts and the GSE53118, which contains only metastasized melanomas, were used to cross-verify prognostic genes described later.

#### 2.1.2. Differential Analysis

To acquire genes differentially expressed between melanoma and normal tissue, expression profiles of control were accessed from the Genotype-Tissue Expression (GTEx) database. Limma analysis was conducted with the absolute value of fold change (FC) set as 2. *p* value less than 0.05 was considered statistically significant.

#### 2.1.3. Immune Infiltration Score

The cytotoxic lymphocyte score calculated by the microenvironment cell populations-counter method (MCP-Counter) was selected as [25] the indicator of cytotoxic lymphocyte infiltration in this study. As a robust quantification of the absolute abundance of cytotoxic lymphocytes, it was used in the weighted gene coexpression network analysis (WGCNA) as each sample's feature to look for closely related gene modules.

#### 2.1.4. WGCNA Analysis and Functional Analyses

For WGCNA analysis, in this study, a minimum module size was set as 30. Modules with eigengene values less than 0.25 were merged into one to present the dendrogram. Hub genes were extracted if their within-module connectivity passed the threshold (module membership > 0.8; gene significance > 0.1; weight > 0.1).

The correlations between module membership from key modules and gene significance of the feature were conducted with Pearson correlation analyses.

Functional enrichment analyses were carried out on the basis of annotations from the Kyoto Encyclopedia of Genes and Genomes (KEGG) with the Database for Annotation, Visualization, and Integrated Discovery (DAVID). The statistically significant threshold was also set as *p* < 0.05.

#### 2.1.5. Protein-to-Protein Interaction Network

With the Search Tool for the Retrieval of Interacting Genes/Proteins (STRING, https://string-db.org/) database, a protein-to-protein network was constructed, and meaningful clusters were identified from it. Interactions of genes in the significant cluster were revisualized with Cytoscape.

### 2.2. Establishment of a Risk-Score Model Based on Genes That Were Prognostic in Melanoma

As mentioned earlier, univariate and multivariate Cox analyses were performed to first identify and verify prognostic genes across the several cohorts involved in this study. Log-rank *p* values with 95% confidence intervals were reported.

Stepwise regression analysis was used to select the optimal risk score model, while the Akaike information criterion (AIC) was used as the evaluation method for the goodness of fit.

### 2.3. Association of the Risk Model with Immune Checkpoint Genes and Responses to Immune Checkpoint Blocker Therapy

Typical immune checkpoint genes, SIGLEC15, TIGIT, CD274, HAVCR2, PDCD1, CTLA4, LAG3, and PDCD1LG2, were selected for comparisons between groups of different levels of risk scores in this study. Mann-Whitney tests were applied for comparisons between two groups under appropriate conditions, and two-tailed *p* values were provided. Bar charts were drawn with the mean ± standard error of the mean (SEM). A *p* value less than 0.05 was considered statistically significant.

Tumor immune dysfunction and exclusion (TIDE) scores were also calculated based on reference [26] for each sample with complete clinical information in TCGA-SKM to predict the possible responses to immune checkpoint blocker therapy. Pearson correlations were conducted to explore the relationships between scores and predict responses.

## 3. Results

### 3.1. WGCNA Analysis Revealed 92 Differentially Expressed Immune-Related Hub Genes That Were Significantly Associated with Cytotoxic Lymphocyte Score

We started with the cohort consisting of 30 primary melanoma samples, which were randomly selected from TCGA-SKM. In the WGCNA analysis, a matrix of immune-related gene expression levels in these 30 samples served as the input. We looked for gene modules significantly associated with cytotoxic lymphocyte scores acquired by MCP-Counter (Figures 1(a) and 1(b)). The brown module was significantly correlated with all major immune cell types, with coefficients ranging from 0.37 to 0.51 (Figure 1(b)), and its module membership scores were also significantly correlated with gene significance for cytotoxic lymphocyte scores (*r* = 0.46, *p* = 1.9*e* − 18, Figure 1(c)). Another module that was much more significantly correlated with cytotoxic lymphocytes was the red module (*p* = 8.3*e* − 3, coefficient 0.47, Figure 1(b)). The module membership scores of this module were also highly positively correlated with the gene significance of cytotoxic lymphocytes (*r* = 0.56, *p* = 3.4*e* − 7, Figure 1(d)). We then conducted differential limma analysis between TCGA-SKM samples (whether primary or metastasized) and normal tissue samples from the GTEx database (Figures 1(e) and 1(f)). We found that among the 92 hub genes, 27 genes were differentially downregulated while 65 genes were upregulated in melanoma samples compared to normal tissue (Figure 1(g)).

We constructed a protein-to-protein network based on the products coded by these 92 genes with the STRING database (average node degree 17.2, average local clustering efficient 0.611, and PPI enrichment value < 1.0*e* − 16) (Figure 2(a)). The pathways these genes were enriched to be significantly related to cell adhesion molecules, Th1 and Th2 cell differentiation, and cytokine-cytokine receptor interactions (Figure 2(b)). According to the MCL clustering (with inflation parameter = 3), there was a major cluster involving 67 genes (average node degree 22.3, average local clustering efficient 0.712, and PPI enrichment value < 1.0*e* − 16) (Figure 2(c)). These genes were enriched to similar functional pathways as the whole list of 92 genes (Figure 2(d)).

### 3.2. Identification of a Signature of 5 Immune-Related DEGs Which Predicted the Prognosis of Melanoma

In order to find if any of the abovementioned genes were related to the prognosis of melanoma, we randomly selected a larger cohort including 69 samples of primary melanoma from TCGA-SKM. In this cohort, univariate Cox analyses were performed for all 67 genes identified from the major cluster of the IR-DEGs highly associated with cytotoxic lymphocyte scores. Genes with log-rank *p* values lower than 0.05 were verified in all TCGA-SKM samples (whether metastasized or not) and validated for the third time in an expression profile including only highly metastasized melanomas (GSE53118). It turned out that 5 genes (CD14, CMKLR1, HCK, ITGB2, and PTAFR) were consistently associated with the prognosis of melanoma, both in primary and metastasized conditions (Table 1); thus, a prognosis model was generated with these 5 genes through multifactor Cox regression based on the survival data available in TCGA-SKM (Figure 3). Using the step function to iterate, in the optimal model (AIC = 2205.157), the risk score of metastasis/poor prognosis was calculated as follows: (−0.02 × expression value of CD14) + (0.1086 × expression value of CMKLR1) + (0.0601 × expression value of HCK) + (−0.3108 × expression value of ITGB2) + (0.0205 × expression value of PTAFR).

Expression patterns of these five genes were consistent between TCGA-SKM and GSE53118 (Figures 3(a) and 4(a)). A higher risk score was significantly associated with a decreased cytotoxic lymphocyte infiltration score (coefficient = −0.62, 95%CI = −0.68 to − 0.56, *p* = 7.22*e* − 50, Figure 3(b)). Furthermore, higher risk scores indicated poorer prognosis, both in mixed primary and metastasized melanoma samples (HR = 2.14, 95%CI = 1.60 to 2.87, *p* = 1.6*e* − 7, Figure 3(c)) and in advanced metastasized samples only (HR = 2.50, 95%CI = 1.39 to 4.48, *p* = 1.5*e* − 3, Figure 4(b)).

### 3.3. Value of the Risk Score in Predicting Responses of Patients with Melanoma to Immune-Checkpoint Blocker Therapy

We examined further how this risk score model indicated a poorer prognosis. Evidence was found from several aspects. First, we chose typical immune checkpoint genes: SIGLEC15, TIGIT, CD274, HAVCR2, PDCD1, CTLA4, LAG3, and PDCD1LG2. The expression levels of these ICGs were compared between high-risk and low-risk groups. Samples that scored high universally expressed significantly low levels of all ICGs we chose (Figures 5(a)–5(h)). We also found that risk scores calculated from this model were significantly related to the infiltration Breslow depth (*p* = 0.0012, Figure 5(i)) and the clinical Clark level of melanoma (*p* = 0.0013, Figure 5(j)).

Considering the low expression levels of immune checkpoint genes in high-risk samples, we predicted the responses of all TCGA-SKM samples to immune checkpoint blocker treatment through the TIDE algorithm (Figure 6). Overall, a weak negative correlation between the risk score from our model and the TIDE score was observed (*r* = −0.14, *p* = 3.5*e* − 3, Figure 6(a)). The correlations between the risk score and TIDE score were analyzed in high-risk and low-risk groups, respectively, and interesting results were observed. Though the coefficient was rather subtle (*r* = 0.14), a higher risk score was associated with a higher TIDE score, i.e., a worse response to immune checkpoint blocker therapy (Figure 6(b)). On the contrary, a comparatively higher risk score in low-risk groups was associated with a significantly lower TIDE score (Figure 6(c)). When the cut-off value was chosen appropriately (Figure 6(d)), the risk score could predict responders well (AUC = 0.711, 95%CI = 0.631 to 0.791).

## 4. Discussion

In the development and progression of melanoma, immunoediting enables cancer cells to escape from the detection and elimination of the adaptive immune system [9]. In a prolonged phase of quiescence, cancer cells are counterbalanced or suppressed because lymphocytes function as the major players in this show [27]. However, some resistant variants of cancer cells are selected during the counterplay with their surrounding microenvironment or peripheral tissues. To continue to survive, they lose or change their immunogenicity, upregulating immune checkpoints and inhibiting immune cells. Immune checkpoint blockers employ this idea to resume the normal function of immune surveillance and elimination to treat malignant melanoma. As early as 2011, a monoclonal antibody targeting cytotoxic T lymphocyte-associated antigen 4 (CTLA-4) called ipilimumab was already approved for metastasized melanoma to recover appropriate cytotoxicity from T cells to kill cancer cells [23, 24]. Monoclonal antibodies such as nivolumab and pembrolizumab target another immune checkpoint axis of the human programmed death 1 (PD-1) receptor with its known death ligands: PD-L1 and PD-L2. Nivolumab delivered a significant effect in prolonging overall survival and progression-free survival compared with dacarbazine in metastasized previously untreated cases [28]. And pembrolizumab exhibited robust effects and achieved a response rate of 24% in patients with advanced disease status even after the ipilimumab regimen [28]. A combination regimen can further demonstrate these therapeutical effects with sustained and confirmed benefits [29]. The MCP-Counter [25] method enabled us to quantify the absolute abundance of cytotoxic lymphocytes from the transcriptomic data of TCGA-SKM. In the first cohort consisting of only primary melanomas, we found that among all the immune-related genes, there were 2 key modules highly related to the infiltration levels of cytotoxic lymphocytes. Most of these hub genes (67 out of 92) were differentially expressed at the overall level among all TCGA-SKM samples. Functional analyses show that these hub genes, along with the major cluster identified within, were tightly associated with differentiation of T lymphocytes, cytokine-to-cytokine receptor interaction, and the functions of cell adhesion molecules. Several models have been developed to predict patient overall survival or general responses to immune checkpoint blockers. Some were generated with integrated machine learning of neural network predictions with clinical data, and some directly encompassed the relations of immune checkpoint genes [26, 30–32]. In accordance with their studies, we also validated the possibility of separating melanoma from the immunologic aspect and the potential of individualized immunotherapies.

In the development of our model, we included genes that were consistently prognostic in different cohorts with heterogeneous samples. This included another cohort selected from TCGA-SKM which only contains primary melanomas, TCGA-SKM itself, and a GSE53118 which contains only highly metastasized melanomas. Besides the association of the risk score calculated from this model with the overall survival, we also associated the risk score with a few histological classifications available. From 1978 to the present, Breslow thickness has remained in all eight editions of the American Joint Committee on Cancer (AJCC) melanoma staging. It has always been consistent in determining the T staging of melanoma and is very reliably prognostic in the newly diagnosed melanoma [33]. Based on the risk score we calculated, TCGA-SKM samples with heterogeneous natures were separated into high-score and low-score groups, and we found that Breslow thickness was significantly higher in samples with higher scores. Another measurement of the invasion depth of melanoma lesions named Clark level was also explored in this study, and a higher invasion level was found to score significantly higher using the prognosis model consisting of five immune-related genes. Even though the Clark level was thought to be less predictive [34], it remained in the AJCC of melanoma staging until it was replaced with the mitotic count in the 7^th^ edition.

There are five genes that were consistently related to the prognosis of melanoma in the cohort we used which is a mixture of primary melanoma lesion samples plus metastasized ones and completely melanoma lesion samples at advanced stages. These genes are CD14, CMKLR1, HCK, ITGB2, and PTAFR.

Monocyte differentiation antigen CD14 has been long suspected to be important in immunomodulation during the pathogenesis of melanoma [35]. CD14 in concert with lipopolysaccharide induces the innate immune responses to bacteria [36–38], and it also leads to NF-kappa-B activation and downstream inflammatory responses. Furthermore, as a vital surface protein for the activation of macrophages, CD14 will be downregulated during the maturation, and dendritic cells are negative for CD14, regardless of the mature situation [35]. High expression of CD14 was confirmed in a study through histochemistry in melanoma samples at advanced stages, while the cells expressing them substantially were suspected to resemble immature monocytes/macrophages [35]. The inflammatory responses arising from the CD14 modulation are crucial clinically in that significant CD14 downregulation was observed in histamine-treated patients with melanoma [35], but the causal relationship is hard to be drawn. Several studies have tried to associate CD14 [39, 40] with the prognosis of melanoma as well as the response to immunotherapy, but the mechanism and the exact role of CD14 in melanoma are not clear. However, it is reasonable to speculate that high expression of CD14 thus will instead be a good standard or signal for better response to treatments [35].

Chemokine-like receptor, CMKLR1, encodes the receptor for the chemoattractant adipokine chemerin/RARRES2. Beyond its function in enhancing adipogenesis and angiogenesis, it also contributes to the reduction of immune responses [41]. Conflicting conclusions have been found across studies of different types of tumors [42–45]; in melanoma mainly, higher levels of chemerin and upregulated CMKLR1 expression have been found to be related to the reduced size of the tumor and increased natural killer cells [46].

HCK encodes the nonreceptor tyrosine-protein kinase that transmits signals from cell surface receptors. It plays a vital role in regulating innate immune responses, including immune cell functions, phagocytosis, cell adhesion, and migration. This kinase also acts with downstream receptors that bind the Fc region of immunoglobulins, receptors in IL-2, IFN-gamma pathway, and integrins, such as ITGB1 and ITGB2. ITGB2 and integrin ITGAL related to ICAM3 contribute to apoptotic neutrophil phagocytosis by macrophages [47]. They also contribute to the natural killer cell cytotoxicity [48]. These two closely associated genes both showed up in our model of predicting responses/prognoses, suggesting that IL-2-related pathways and the function of macrophages are important in melanoma. But the application of ibrutinib, a drug that targets IL-2 inducible kinase (which is highly expressed in melanoma), did not deliver any clinical benefits in patients with metastatic melanoma whose PD-1 treatment was failed [49]. Our model provided more insights into this by revealing another inflammation-related gene indicative of immunotherapy response and closely related to the prognosis: PTAFR. It is a receptor for platelet-activating factor, a chemotactic phospholipid mediator that possesses potent inflammatory activity. It has been demonstrated that the failure of chemotherapeutic processes in melanoma resulted in a PTAFR-dependent fashion and the tumor growth was augmented. The oxidative stress that came along with the activation of PTAFR induced damage to the immune system [50, 51]. In mouse melanoma tumor models, voluntary exercise may ameliorate the immune response and inflammatory response in lesion sites with PTAFR as one of the hub genes in regulating oxidative pathways and complement pathways [52]. Interestingly, the integrins mentioned above such as integrins ITGAM/ITGB2 and ITGAX/ITGB2 are also receptors for the iC3b fragment of the third complement component and for fibrinogen.

In this study, samples in the low-risk group universally expressed significantly high levels of several known immune checkpoint genes, such as SIGLEC15, TIGIT, CD274, HAVCR2, PDCD1, CTLA4, LAG3, and PDCD1LG2. Furthermore, according to this result, the model score is negatively correlated with the TIDE score, indicating a higher possibility of immune checkpoint blocker therapy in the low-risk group than that in the high-risk group. Resistance to immune checkpoint blockers is a considerable barrier and challenging problem in exploiting immunotherapies in advanced patients with melanoma. Little is known about the exact mechanisms of primary or secondary resistance, but low expression of immune checkpoint genes at baseline tumor tissue has been hypothesized to be the reason for primary resistance [53]. Based on this, we suspect that there could be two subsets in the high-risk group identified through this model: either they are expressing low levels of immune checkpoint genes in nature, and not responding to any ICB due to this reason, or they have not developed their ways of immunoediting yet, i.e., they have not started to highly express specific ICGs to counteract with the defenses from the immune system. If they begin to do so, it is highly likely that they will be responsive to that particular ICB therapy. However, there is a lack of specific cellular and animal experiments for validation, and further in vivo and ex vivo experiments are needed for future improvement.

## Figures and Tables

**Figure 1:** 92 differentially expressed immune-related hub genes were significantly associated with cytotoxic lymphocyte infiltration scores in melanoma samples. (a) Hierarchical dendrogram of WGCNA; (b) correlation heatmap of infiltration scores from the MCP-Counter algorithm with modules; (c, d) scatterplot of gene significance of cytotoxic lymphocyte score versus (c) brown and (d) red module membership; (e, f) volcano plot and expression heatmap presenting the results of differential analysis between melanoma and normal tissue; (g) Venn plot of differentially regulated genes and hub genes that are significantly correlated with the infiltration score of cytotoxic lymphocytes.

**Figure 2:** Predicted protein interactive network constructed based on hub genes and key enriched pathways. (a, b) Network of 92 IR-DEGs after MCL clustering and significant pathway they enriched into; (c, d) network of 67 genes in the major cluster and significant pathway they enriched into.

**Figure 3:** Efficacy of the 5-IR-DEG risk model in predicting overall survival of TCGA-SKM. (a) Risk score distribution, survival status of all samples, and expression heatmap of five genes; (b) correlation of the risk score and infiltration score of cytotoxic lymphocytes; (c) Kaplan-Meier survival of this prognostic model in TCGA cohort.

**Figure 4:** Efficacy of the 5-IR-DEG risk model in GSE53118. (a) Risk score distribution, survival status of all samples, and expression heatmap of five genes; (b) Kaplan-Meier survival of this prognostic model in GSE53118.

**Figure 5:** High immune-related model scores indicated low expression levels of classic immune checkpoint genes and deep infiltration in the primary tumor site. (a–h) Comparisons of expression levels of CD274, CTLA4, HAVCR2, LAG3, PDCD1, PDCD1LG2, SIGLEC15, and TIGIT between the low-score group and the high-score group; (i) comparison of the Breslow depth between the low-score group and the high-score group; (j) comparison of the score between the low Clark level (I and II) group and the high Clark level (III to V) group.

**Figure 6:** Association of the 5-IR-DEG risk model and predicted responses to immune checkpoint blocker therapy. (a) Overall correlation between model score and TIDE score; (b) correlation between model score and TIDE score in the high-risk group; (c) correlation between model score and TIDE score in the low-risk group; (d) ROC curve when using the model score to predict responders of low-risk subjects.

**Table 1:** Results of univariate Cox analyses.

Gene	Cohort 2: 69 samples of primary melanoma				All TCGA-SKM samples				GSE53118: 79 metastasized melanoma samples			
	HR	Low 95% CI	High 95% CI	Log rank	HR	Low 95% CI	High 95% CI	Log rank	HR	Low 95% CI	High 95% CI	Log rank
CD14	1.00540	1.00039	1.01043	0.02970	0.58732	0.44774	0.77042	0.00012	0.73561	0.56706	0.95424	0.01956
CMKLR1	1.15676	1.01574	1.31737	0.02402	0.62832	0.47988	0.82269	0.00073	0.38604	0.17158	0.86857	0.01976
HCK	1.06897	1.01007	1.13130	0.01867	0.53355	0.40626	0.70074	0.00001	0.64748	0.44118	0.95023	0.02515
ITGB2	1.02357	1.00469	1.04280	0.01090	0.55908	0.42627	0.73328	0.00003	0.77982	0.61092	0.99541	0.04441
PTAFR	1.11806	1.03635	1.20622	0.00231	0.60681	0.46314	0.79504	0.00029	0.33987	0.14557	0.79352	0.01181

## Data Availability

The bioinformatics data supporting this bioinformatics analysis are from previously reported studies and datasets, which have been cited. The processed data are available TCGA and GEO database.
